The article "An AI-Driven Hybrid Framework for Intrusion Detection in IoT-Enabled E-Health" was retracted in 2023. Reasons: signs of a paper mill; compromised peer review; unreliable results or conclusions.

# An AI-Driven Hybrid Framework for Intrusion Detection in IoT-Enabled E-Health

**DOI:** 10.1155/2022/6096289

**Published:** 2022-08-21

**Authors:** Fazal Wahab, Yuhai Zhao, Danish Javeed, Mosleh Hmoud Al-Adhaileh, Shahab Ahmad Almaaytah, Wasiat Khan, Muhammad Shahid Saeed, Rajeev Kumar Shah

**Affiliations:** ^1^College of Computer Science and Technology, Northeastern University, Shenyang 110169, China; ^2^Software College, Northeastern University, Shenyang 110169, China; ^3^Deanship of E-Learning and Distance Education, King Faisal University, P.O. Box 400, Al-Ahsa, Saudi Arabia; ^4^Applied College in Abqaq, King Faisal University, Al-Ahsa, Saudi Arabia; ^5^Department of Software Engineering, University of Science and Technology Bannu, Bannu, Pakistan; ^6^Dalian University of Technology, Dalian 116024, China; ^7^Sunway International Business School, Kathmandu, Nepal

## Abstract

E-health has grown into a billion-dollar industry in the last decade. Its device's high throughput makes it an obvious target for cyberattacks, and these environments desperately need protection. In this scientific study, we presented an artificial intelligence (AI)-driven software-defined networking (SDN)-enabled intrusion detection system (IDS) to address increasing cyber threats in the E-health and internet of medical things (IoMT) environments. AI's success in various fields, including big data and intrusion detection systems, has prompted us to develop a flexible and cost-effective approach to protect such critical environments from cyberattacks. We present a hybrid model consisting of long short-term memory (LSTM) and gated recurrent unit (GRU). The proposed model was thoroughly evaluated using the publicly available CICDDoS2019 dataset and conventional evaluation measures. Furthermore, for proper validation, the proposed framework is compared with relevant classifiers, such as cu-GRU+ DNN and cu-BLSTM. We have further compared the proposed model with existing literature to prove its efficacy. Lastly, 10-fold cross-validation is also used to verify that our results are unbiased. The proposed approach has bypassed the current literature with extraordinary performance ramifications such as 99.01% accuracy, 99.04% precision, 98.80 percent recall, and 99.12% F1-score.

## 1. Introduction

The internet of things (IoT) has been identified as an essential research domain for the present and coming decade. The applications of IoT have been integrated into industries and health areas to aid the people and emerged as industrial internet of things (IIoT) and IoMT. The IIoT revolution is exploding, resulting in massive monetary gains and automation [1]. On the other hand, the IoMT has also grown into a multibillion-dollar industry. While providing significant benefits, the pervasive and open nature of the IoMT ecosystem makes it a possible target for various emerging cyber threats and attacks [2–5]. The extensive connectivity and continuous sharing of data of these devices make them a prime target of different threat actors that can execute anomalous activities against them [6]. The exploit's motivations are to obtain important information, steal money, and damage the system's resources [7–9]. As the number of linked IoT devices grows, critical infrastructure and assets of different organizations are also becoming vulnerable to numerous cyberattacks. Cyber threats could cost up to $ 90 trillion by 2030 if no reasonable alternative is given before then [10, 11]. IoMT environments pose three issues as follows: The first is the heterogeneous network and dynamic nature, the second is its hugely scattered design, and the last is the protocols that the IoT use to address concerns like computing limits and power consumption in network sensors [12, 13]. The most common issue in IoMT setups is keylogging, botnet attacks, and zero-day exploits [14–16].

The article "An AI-Driven Hybrid Framework for Intrusion Detection in IoT-Enabled E-Health" was retracted in 2023. Reasons: signs of a paper mill; compromised peer review; unreliable results or conclusions.

The intruder's primary purpose is to contaminate sensitive machines with different techniques, including denial-of-service (DoS) attacks, distributed denial of service (DDoS), and advanced persistent threats (APTs), in order to gain control and change their functioning [17, 18]. The nuclear program of Iran, for example, was targeted by the Stuxnet worm in 2010. Later, in 2013, Iranian hackers gained access to the dam's ICS. In Ukraine, Black Energy malware caused a power outage for 230,000 people in 2015 [19]. As a result, these incidents demonstrated that typical cybersecurity methods, such as authentication, security rules, security firewalls, both software and hardware-based, and IDS, are no longer beneficial.

Similarly, the IIoT's digital landscape is vulnerable to sophisticated hacking techniques, physical security risks, and a wide range of devices that can be easily infected by botnet attacks [20]. Furthermore, the IoMT demands a different detection mechanism for its environments due to low latency and resource limitations. Hence, such environments need a scalable, cost-effective, and adaptive intrusion detection mechanism against emerging cyber threats. The proposed network model is shown in Figure 1.

### 1.1. Contribution

The main contributions of this research are as follows:

- We presented a novel, i.e., Cu-LSTM+ GRU SDN-enabled intelligent framework to detect threats quickly and effectively in the IoMT environment. The proposed SDN-enabled model does not overburden the IoMT resource.
- We employed a publicly available, state-of-the-art CICDDoS2019 dataset to evaluate the performance of the proposed model.
- We evaluated the proposed model's performance by employing two existing benchmark algorithms, i.e., Cu-GRU-DNN and Cu-BLSTM, which were trained and assessed on the same dataset.
- To comprehensively assess the proposed model's performance, we have compared it to the existing literature.
- For a better assessment, we have utilized the standard evaluation metrics.
- Finally, 10-fold cross-validation is also used to verify that our results are unbiased.

The article "An AI-Driven Hybrid Framework for Intrusion Detection in IoT-Enabled E-Health" was retracted in 2023. Reasons: signs of a paper mill; compromised peer review; unreliable results or conclusions.

The rest of this paper is organized as follows: the background and existing literature are explained in Section 2. The proposed approach, dataset, and other specifics are discussed in Section 3. Experimentation and assessment criteria are covered in Section 4.  Section 5 consists of results and discussion. Finally, the conclusions and future work of this research are given in Section 6.

## 2. Background and Existing Literature

In the years ahead, SDN is likely to be the most promising networking model. An application plane, data plane, control plane, and respective APIs, i.e., southbound API and northbound API, make up SDN's architecture. The communication between the applications and controller is based on the northbound interface. The functions of the southbound APIs include communicating with network virtualization protocols, switching fabric, and also a decentralized computing network. The SDN architecture separates the control plane from the application and data plane [8]. The control plane is a centralized and intelligent device that gives an overview of the underlying network. In addition, the control plane is a concentrated data processing and decision-making unit. It also can send data across the entire network. The data plane, on the other hand, represents the collection of SDN agents and the devices used for forwarding. Because the whole framework is dependent on the control plane, it is configurable and has the ability to expand its capabilities by incorporating further modules. As a result, SDN offers flexibility and creativity, and its detailed design is explained in [21]. All SDN controllers can extend different modules.

Because of this, the authors' proposed detection technique is implemented on the control plane. The architecture and design of different SDN controllers are mostly the same; nevertheless, their functionality differs. The implementation language varies from controller to controller. Floodlight, for example, uses Java as its implementation language, while POX is written in Python. According to modern scientific evolution, the IoT has manifested competencies that touch almost every aspect of our life. Because of its ease of acquisition, IoT is vulnerable to a variety of security threats that must be handled. SDN is a powerful technology that offers a potential way out for IoT security and integrity.

The article "An AI-Driven Hybrid Framework for Intrusion Detection in IoT-Enabled E-Health" was retracted in 2023. Reasons: signs of a paper mill; compromised peer review; unreliable results or conclusions.

In the past few years, scholars have shown a keen interest in DL and its applicability in a variety of fields, including vehicle production, law, and health care [22–24]. The DL techniques have improved the area of computer engineering through various applicabilities, which are practically employed in every industry, from medical appliances to self-driving cars. The deep neural network (DNN) models make use of the neural network architecture, which is why they are termed as deep neural networks [25–27]. These models are trained on a large amount of labeled data and to extract features from it without the need for human intervention. Additional DL applications include speech recognition software, fraudulent activity detection, image categorization, and intrusion detection. It can also be used to detect pedestrians, which reduces accidents. Different technological efforts have been made to address IoT's vulnerable characteristics; nevertheless, SDN-based security solutions have shown to be the most effective [28]. Other cutting-edge technologies link with SDN to effectively fulfill the purpose under issue. The SDN blockchain integration is shown, which addresses all of the critical security apprehensions of IoT from an ultramodern standpoint. The primary ability of that amalgamation is the protection from DoS attacks, impersonating attacks, and routing attacks [29–32]. Furthermore, there is a lot of effort in the field of NIDS in SDN [33]. Another security model that should be discussed here is designed to protect the critical IoT ecosystem from many types of security attacks. The proposed scheme is a large-scale responsive atmosphere SDN-enabled blockchain-inspired solution. The model's performance is examined, and the positive results appear to make it an appropriate alternative for large-scale IoT networks [34]. SDN collaborates with the convolutional neural networks (CNN) to provide notable protection for IoT against a wide range of genuine issues. The tree of DDoS-based attacks is a warning indicator that communication in an IoT-based autonomous ecosystem may be disrupted. This behavior attracted the concentration of researchers, prompting the creation of an SDN-enabled CNN-based security architecture for IoT networks with limited resources. The proposed framework's most notable attribute is its ability to detect security threats quickly while using minimal network tools [7].

In terms of resource consumption, SDN-enabled security systems are thought to be outstanding. The SDN central controller's constitutional scheduling mechanism is always accompanied by exceptional network resource management. As a result, the attribute is passed down to SDN-enabled intrusion detection techniques, making it easier for IoT to satisfy defense frameworks while using the fewest resources possible [35]. In reference [36], the researchers presented a biometric mechanism to improve IoT security. The security of the system has been increased by an average of 96.82% using the suggested methodology. They used a combination of biometrics and coding. Based on experimental results, the given solution enhances the security of the system by an average of 120.38%. By using biometric features and incorporating the findings of the evaluation, the risk of potential security issues occurring is reduced by 90.71%. Furthermore, because of IoT-specific service requirements (i.e., resource restrictions, low latency, flexibility, dissemination, and portability), attack detection differs dramatically from the previous approaches [36]. As a result, an adjustable, modular, dynamic, and cost-effective detection method against a variety of prevalent emerging cyber threats is critical for the IoMT networks. The authors of [37] used GRU-RNN for NIDS. They used the NSL-KDD dataset with six basic features and obtained an accuracy of 89%, which is insufficient for today's emerging security attacks.

The article "An AI-Driven Hybrid Framework for Intrusion Detection in IoT-Enabled E-Health" was retracted in 2023. Reasons: signs of a paper mill; compromised peer review; unreliable results or conclusions.

In reference [38], an IoT-enabled healthcare system prototype-based framework is given. The solution makes use of a smart gateway design to make data storage and processing easier, and cloud-based analysis and decision-making. The security of this solution is determined by the operating system's security features and capabilities. The authors of [39] proposed a deep learning-based technique for detecting anomalies. CNN, LSTM, and MLP were employed in this system. Tshark and Wireshark were used to collect data for the experiment. In reference [40], the hierarchical architecture for usage in the domain of health is discussed, and the security of the data. Information relating to health data analysis is maintained separately in the cloud and fog infrastructure in this way. The MAPE-K-based model is also used in the solution to provide computations for executing various applications along with data encryption. In reference [41], the researchers suggested a DL technique for flow-based intrusion based on a DNN. This framework used Snort (a network intrusion detection system) and Barnyard and obtained 85% accuracy. The authors of [42, 43] proposed a technique in SDN that relies on multilayer perception to overcome concerns with the botnet detection mechanism (MLP). Real data were used in the experiment, with a 98% accuracy rate. The authors proposed an RNN-based IDS in [44, 45] and used the NSL-KDD dataset for training. The analysis was carried out on the network traffic. For multiclass classification, this approach secured an accuracy rate of 81.29%. In reference [46], the authors described an intelligent SDN-based method for IoT intrusion detection. The researchers trained and experimented with deep learning classifiers on the CICIDS2017 dataset and improved detection accuracy.

The article "An AI-Driven Hybrid Framework for Intrusion Detection in IoT-Enabled E-Health" was retracted in 2023. Reasons: signs of a paper mill; compromised peer review; unreliable results or conclusions.

## 3. Materials and Methods

This paper proposed an intelligent DL-driven threat detection technique for IoMT scenarios. This part covers our research approach, including the hybrid attack architecture, dataset description, proposed detection model, environmental setup, and metrics used for evaluation.

### 3.1. Detection Technique and Network Model

The SDN has grown in popularity as an embedded design during the last few years. The application plane of the SDN is designed to operate a wide range of apps and supply various services to end users. The control plane and the data plane are separated in the SDN design for simplicity and flexibility. On the other hand, the SDN's control plane is in charge of transmitting data, routing selections, and threat detection. Furthermore, the control plane improved the network's global view and main controller capabilities, making the collection of network data easier. To detect risks and exploitation in the IoMT environment, we propose Cu-LSTM+ GRU. The proposed model is placed in the SDN control plane, as shown in Figure 1. It is placed in the control plane for a variety of motives.

First and foremost, it is fully programmable and can also extend IoMT devices on the data plane. Second, SDN provides a solution for heterogeneity among IoMT devices and SDN controllers. Furthermore, the control plane can manage the primary IoMT devices in its data plane without depletion. The data plane is responsible for transporting data packets from the source to the destination and forwarding actual IP packets. The SDN framework and IoMT integration present a better solution to thoroughly monitor network traffic to detect intrusions, unauthorized events, and security attacks while being cost-effective and centrally controlled.

The Cu-LSTM+ GRU model is used in this strategy to detect advanced malware in the IoMT scenario. With better detection ratios and minimal false positives, the training and testing of the proposed model are performed by using the CICDDoS 2019 dataset. The proposed model consists of multiple layers, i.e., LSTM consists of 3 hidden layers with 600, 400, and 200 neurons while GRU consists of 2 layers of 300 and 150 neurons, respectively. For the activation function in the output layer, we employed softmax and ReLU in the other layers. The experimentation was carried out using 64 batch sizes until 20 epochs for better outcomes. The experiment is performed with the CUDA-enabled version. Furthermore, the proposed approach makes use of TensorFlow's backend and Python's Keras framework. A comparison is made with the proposed approach using the two classifiers. Cu-GRU+ DNN consists of 2 layers of GRU and 2 layers of DNN with 400, 300, 300, and 100 neurons. However, Cu-BLSTM has three layers with neurons of 400, 300, and 100, respectively.

The article "An AI-Driven Hybrid Framework for Intrusion Detection in IoT-Enabled E-Health" was retracted in 2023. Reasons: signs of a paper mill; compromised peer review; unreliable results or conclusions.

### 3.2. Dataset

The selection of an adequate dataset is critical when evaluating the performance of threat detection schemes. The literature research reveals that different authors used different datasets for threat identification in such environments, such as NSL-KDD, KDD CUP99, and so on. Many of them lack the IoT support feature. Hence, the proposed work used an IoT-based dataset, i.e., CICIDDoS2019 [47], which is publicly available. This dataset contains the most serious malware, such as DDoS and reflection attacks. Furthermore, the dataset is based on network flow and has IoMT supporting characteristics. The dataset contains more than 80 traffic features. The proposed model is concerned with 9 classes of the dataset. The details of the attacks and their instances are given in Table 1.

### 3.3. Dataset's Preprocessing

The following steps were used to preprocess the dataset in the proposed study. We initially identified all rows with NaN values and blank rows and further eliminated them completely, so the proposed model's performance and quality of data may not be affected. Using the label encoder, we next make the numeric values from all the non-numeric values, i.e., sklearn, because the DL algorithms mostly interpret numeric data. In addition, we used one-hot encoding on the output label to limit the odds of unexpected results, as model performance can be affected by category sorting. For data normalization, we used the MinMaxScaler, which improves the model's efficiency.

## 4. Environment/Experimental Setup

In our experiment, we used a graphic processing unit (GPU) and a Core i7-7700 processor for testing purposes. Furthermore, Python V3.9 and Keras have been used to train the suggested module. The experiment requirements, such as hardware and software requirements, are listed in Table 2.

### 4.1. Metrics Used for Evaluation

We assessed the suggested architecture's performance using standard assessment measures such as precision, recall, accuracy, and F1-score. In order to determine specific values (MCC), we have to calculate the true positive (TP), true negative (TN), false positive (FP), false negative (FN), false omission rate (FOR), and Matthew's correlation coefficient.

The article "An AI-Driven Hybrid Framework for Intrusion Detection in IoT-Enabled E-Health" was retracted in 2023. Reasons: signs of a paper mill; compromised peer review; unreliable results or conclusions.

## 5. Results and Discussion

In this section, we have described the complete results of our proposed hybrid model (Cu-LSTM+ GRU). We also compared this model against two additional hybrid models, i.e., Cu-GRU+ DNN and Cu-BLSTM, and current methodologies in the literature, for a thorough performance review. The authors also performed a 10-fold cross-validation to show the unbiased results of the proposed model. The results are given in Table 3. Furthermore, the performance of our proposed model is assessed with the help of the standard metrics mentioned below.

### 5.1. ROC Curve Analysis

The effectiveness of an IDS can be evaluated using the critical metric known as ROC. True-positive (TPR) and true-negative (TNR) rates are associated, and the findings are plotted using ROC. The ROC curve for our approach is shown in Figure 2. The link between a true positive and a true negative is depicted in the following diagram. The figure depicts the efficacy of the proposed model.

### 5.2. Confusion Matrix Analysis

The classification model's output is shown in this evaluation matrix. The proposed model Cu-LSTM+ GRU accurately recognizes the classes based on the confusion matrix results.  Figure 3 shows the confusion metrics for the proposed models proving that it successfully identifies the classes correctly and efficiently.

### 5.3. Precision, Recall, Accuracy, and F1-Score

The accuracy of a classifier demonstrates its efficiency and performance [48]. It indicates how many samples the suggested technique correctly identifies. The accuracy performance of the proposed model is shown in Figure 4. This hybrid model has a 99.01% accuracy rate and a 98.80% recall rate. The records that are accurately identified reflect precision.

Furthermore, our suggested model has a precision of 99.04% and an F1-score of 99.12%, respectively. Complete detail of each fold is also given in Table 2 regarding the accuracy and other evaluation metrics. The per-class accuracy of all the three models is also provided in Table 4, proving the efficiency of the proposed model.

### 5.4. FDR, FPR, FNR, and FOR Analysis

We calculated the FDR, FOR, FPR, and FNR to adequately examine our proposed technique.  Figure 5 shows the results. The FOR and FPR of Cu-LSTM-GRU have a value of 0.00172% and 0.00193%, whereas FNR and FDR are 0.00121% and 0.00164%, respectively. As a result, the proposed model, i.e., Cu-LSTM+ GRU, outperforms the other two models. Furthermore, Cu-GRU+ DNN shows better performance than Cu-BLSTM.

The article "An AI-Driven Hybrid Framework for Intrusion Detection in IoT-Enabled E-Health" was retracted in 2023. Reasons: signs of a paper mill; compromised peer review; unreliable results or conclusions.

### 5.5. MCC, TNR, and TPR Analysis

To further assess the proposed model, we employed a confusion matrix to conduct an in-depth study of the MCC, TNR, and TPR analysis results. MCC, TNR, and TPR have values of 98.92%, 99.36%, and 99.13%, respectively. A closer examination of Figure 6 demonstrates that the proposed model outperforms the other two models.

### 5.6. Speed Efficiency

The testing time taken by our suggested method is demonstrated in Figure 7. We do not include the training phase because it was primarily performed offline. Testing is crucial when demonstrating the model's performance and efficiency. Our suggested hybrid techniques took only 19.35 ms to complete, which is a computationally efficient time. Cu-BLSTM, on the other hand, is computationally superior to Cu-GRU-DNN, having a testing time of 24.50 ms.

### 5.7. The Comparison of Cu-LSTM+ GRU with the Existing Literature

We compared the proposed method with the existing two hybrid DL models (Cu-GRU+ DNN and Cu-BLSTM) to demonstrate its efficacy. Both models were evaluated using the same metrics and dataset, and the CICDDoS2019 dataset has been used to test and train all three models.

A comparison with other benchmark algorithms is also made.  Table 5 shows a comparison of the suggested model to the current literature. The proposed model (Cu-LSTM+ GRU) clearly surpasses the existing literature regarding the accuracy, F1-score, precision, and speed efficiency. In addition, the suggested model's testing time is only 19.35 ms, which is much faster than previous benchmarks.

## 6. Conclusions and Future Work

With the development of IoMT and E-health, the risk of cyber assaults has skyrocketed. These diverse devices make deploying traditional intrusion detection systems challenging in such environments. Therefore, the SDN paradigm provides a promising solution for protecting IoMT/E-health infrastructures. The proposed framework provides a quantitative, economical, and precise solution. A complete model test is run in combination with typical test metrics. We compared the result of the proposed model with two other classifiers that have been trained and evaluated under the same environment and with the current benchmarks. The proposed hybrid Cu-LSTM+ GRU model outperforms the current benchmark models with 99.01% accuracy and precision and F1-score of 99.12% and 99.04%, respectively. Furthermore, the computational complexity of the proposed model is very low, i.e., 19.35 ms. Despite its great performance, our proposed technique has a shortcoming that we intend to solve in the future, i.e., the proposed model would be more beneficial if it could identify insider threats.

The article "An AI-Driven Hybrid Framework for Intrusion Detection in IoT-Enabled E-Health" was retracted in 2023. Reasons: signs of a paper mill; compromised peer review; unreliable results or conclusions.

In the future, we aim to use some other deep learning algorithms with blockchain to develop a new intrusion detection system for such environments. Finally, the authors endorse SDN-empowered, deep learning-based intrusion detection systems for the security of IoMT environments.

## Figures and Tables

**Figure 1:** Proposed SDN-based model.

**Figure 2:** ROC curve of LSTM+ GRU.

**Figure 3:** Confusion matrix of cu-LSTM+ GRU.

**Figure 4:** Overall comparison of the proposed model against Cu-GRU+ DNN and Cu-BLSTM.

**Figure 5:** FPR, FNR, FDR, and FOR of the models.

**Figure 6:** TPR, TNR, and MCC of the models.

**Figure 7:** Testing time of Cu-LSTM + GRU, Cu-GRU + DNN, and Cu-BLSTM.

**Table 1:** CICDDoS 2019 details.

Attacks	Instances
Normal	56,600
DrDoS-MSSQL	2400
Dr-DoS	2350
DrDoS-SSDP	2368
PORTMAP	2496
UDP-lag	2300
SYN	2341
DrDoS-UDP	2600
WebDDoS	2365
Total	**75,820**

**Table 2:** Experimental setup.

Processor	I7 (3.33 GHz)
OS	Windows 10
RAM	16 GB
Language	Python
GPU	Geforce 1060
IDE	Spyder
Generation	8^th^
Libraries	NumPy, TensorFlow, pandas, Keras, and scikit-learn

**Table 3:** 10-Fold results of Cu-LSTM+ GRU, Cu-GRU+ DNN, and Cu-BLSTM.

	Model	1	2	3	4	5	6	7	8	9	10
Accuracy (%)	Cu-LSTM+GRU	98.25	98.23	99.15	98.89	99.08	99.31	99.16	99.12	99.16	99.84
	Cu-GRU+DNN	97.56	97.21	97.86	97.54	98.54	98.57	99.15	98.81	98.62	98.86
	Cu-BLSTM	98.36	98.36	98.41	98.93	98.87	98.87	98.69	98.36	98.24	98.29

F1-score (%)	Cu-LSTM+GRU	98.24	98.63	99.68	99.06	99.06	99.25	99.19	99.34	99.08	99.68
	Cu-GRU+DNN	98.62	98.45	98.15	98.62	98.62	98.74	99.11	99.15	98.82	98.18
	Cu-BLSTM	98.94	98.91	98.29	98.29	98.68	98.15	98.19	98.81	99.16	99.43

Recall (%)	Cu-LSTM+GRU	98.96	98.92	99.26	98.61	98.21	98.61	98.89	98.97	98.69	98.92
	Cu-GRU+DNN	98.15	98.06	98.04	98.04	98.61	98.25	98.54	98.95	99.15	98.87
	Cu-BLSTM	98.15	98.16	98.16	98.85	98.71	98.06	98.15	98.64	98.64	98.86

Precision (%)	Cu-LSTM+GRU	98.16	98.68	99.14	99.14	99.32	99.36	99.86	99.51	98.91	98.34
	Cu-GRU+DNN	98.69	98.85	98.85	98.09	97.93	97.19	98.14	98.31	98.16	98.31
	Cu-BLSTM	98.19	98.96	98.48	98.48	98.86	98.46	98.69	99.05	99.17	98.78

**Table 4:** Per-class accuracy of the models.

Class	Cu-LSTM+GRU	Cu-GRU+DNN	Cu-BLSTM
Normal	99.84	98.86	98.93
DrDos-MSSQL	98.15	97.56	98.87
DrDoS-SSDP	99.12	98.54	98.29
DrDoS	98.23	97.86	98.36
SYN	98.25	97.21	98.24ss
WebDDoS	99.16	98.57	98.36
PORTMAP	99.31	99.15	98.93
DrDoS-UDP	99.08	98.62	98.41
UDP-lag	99.15	98.81	98.87

**Table 5:** Comparison with the existing literature.

Ref	Model	Accuracy (%)	Recall (%)	F1-score (%)	Precision (%)
Proposed	Cu-LSTM+ GRU	99.01	98.80	99.12	99.04
[49]	GRU-RNN	89.00	91.00	92.50	94.00
[17]	CNN	91.50	—	—	—
[50]	GRU-LSTM	87.90	77.90	80.60	83.50

The article "An AI-Driven Hybrid Framework for Intrusion Detection in IoT-Enabled E-Health" was retracted in 2023. Reasons: signs of a paper mill; compromised peer review; unreliable results or conclusions.

## Data Availability

Since the funding project is not closed and related patents have been evaluated, the simulation data used to support the findings of this study are currently under embargo while the research findings are commercialized. Requests for data, based on the approval of patents after project closure, will be considered by the corresponding author.
